# Shrunken Pore Syndrome Is Associated with Renal Function Decline in Female Patients with Kidney Diseases

**DOI:** 10.1155/2022/2177991

**Published:** 2022-07-07

**Authors:** Zhongcai Wu, Le Wang, Yueqiang Li, Ying Yao, Rui Zeng

**Affiliations:** ^1^Department of Nephrology, Tongji Hospital, Tongji Medical College, Huazhong University of Science and Technology, Wuhan 430030, China; ^2^Department of Nutrition, Tongji Hospital, Tongji Medical College, Huazhong University of Science and Technology, Wuhan 430030, China

## Abstract

**Background:**

Shrunken pore syndrome (SPS) represents selective impairment of kidney filtration of low-molecular-weight molecules between 1 and 30 kDa and has been related to outcomes including morbidity, mortality, and cardiovascular events. However, the prevalence and kidney outcomes of SPS have not been investigated in patients with IgA nephropathy (IgAN) and membranous nephropathy (MN).

**Methods:**

We retrospectively collected information of 536 patients including 414 with IgAN and 122 with MN. SPS was mainly defined by cystatin C-based eGFR < 70% of creatinine-based eGFR using the CAPA-LM equation pairs, while CKD-EPI equations were also employed in sensitivity analyses. Prevalence rate of SPS and its association with end-stage renal disease (ESRD) or severe eGFR decline (≥50% eGFR reduction or doubling of baseline creatinine) were investigated.

**Results:**

44% (8%) patients were identified as possessing SPS using the CAPA-LM definition. ESRD happened in 24 patients during the average follow-up period of 27.7 months. Despite dramatic increase of incidence rate of ESRD for SPS, significant hazard ratio (HR) only existed in IgAN patients after multivariable adjustment (HR: 8.35, 95% CI: 2.10~33.26), but lost significance in sensitivity analyses. 36 patients were determined as having experienced severe eGFR decline after excluding transient creatinine fluctuation. SPS was associated with severe eGFR decline by Kaplan-Meier survival analyses in the overall population as well as the IgAN, MN, male, and female subpopulations, which remained significant in multivariable adjustments in all groups except IgAN. However, only in female patients the association between SPS and eGFR decline remained significant in all the sensitivity analyses.

**Conclusions:**

SPS was independently associated with eGFR decline in female patients with IgAN and MN.

## 1. Introduction

The kidneys are important organs governing fluid homeostasis and substance excretion. Reduced kidney function has become prevalent and is devastating as it greatly increases morbidity, mortality, and cardiovascular complications [1]. Current evaluation of kidney function mainly involves the assessment of glomerular filtration rate (GFR), which represents the volume filtered through the glomerular filtration barrier per unit of time. Conventional methods for GFR assessment measure the filtration of small molecules below 1 kDa with sieving coefficients close to 1, such as inulin, 99Tc-DTPA, and creatinine [2].

However, the role of kidney is far beyond the filtration of small molecules. A substantial proportion of low-molecular-weight molecules within 1~30 kDa are cleared by kidneys in normal physiology, but this function has long been overlooked among academic society [3–5]. Cystatin C (13.3 kDa) represents a characteristic protein that is mainly excreted by kidneys [6], and corresponding equations have been developed to evaluate GFR [7, 8]. Under certain pathological statuses where the glomerular filtration pores shrink [9] or glomerular filtration membrane thickens [10], the filtration of low-molecular-weight proteins could be selectively impaired while filtration of small molecules are almost unchanged. This phenomenon has been noted recently and tentatively termed as “shrunken pore syndrome (SPS),” which is defined by cystatin C-based estimation of eGFR (eGFRcys) being less than 60% or 70% of creatinine-based estimation of eGFR (eGFRcr) [11, 12].

So far, SPS has been identified in diverse populations from pregnant women [9] to patients with heart failure [13], hip fracture [14], undergoing cardiac surgery [15, 16], and even seemingly healthy ones [17, 18]. Detrimental health effects have been characterized in almost all related researches concerning various outcomes such as morbidity [17], mortality [13, 16], rehospitalization [13], and cardiovascular events [19, 20]. Yet, SPS has rarely been investigated in patients with kidney diseases, and its relation to renal outcomes has not been clearly elucidated. To clarify this issue, we conducted this retrospective cohort study focusing on SPS and its relationship with renal outcomes in patients with biopsy-proven IgA nephropathy (IgAN) and membranous nephropathy (MN).

## 2. Materials and Methods

### 2.1. Study Design

This is a retrospective cohort study based on subjects with biopsy-proven IgAN or MN admitted to Tongji Hospital between December 2011 and September 2019. The study was approved by the medical ethical review board of Tongji Hospital, Tongji Medical College, Huazhong University of Science and Technology, and was conducted according to the Declaration of Helsinki. Informed consent was waived due to its retrospective design and observational nature.

### 2.2. Study Population

1741 patients with IgAN and 650 patients with MN were screened, and those were included with simultaneous measurements of cystatin C and creatinine at baseline when corticosteroids were not used. Patients who were pregnant, less than 18 years old, undergoing renal replacement therapy, with AKI, uncontrolled malignant neoplasm, thyroid diseases, end-stage renal disease (ESRD), syphilis, adrenal cortical insufficiency, concomitant ANCA vasculitis, or SLE were excluded. The final sample enrolled 536 patients.

### 2.3. Data Collection

We collected information on kidney pathology from biopsy records and demographic, behavioral, and laboratory information together with data on comorbidities and medications from electronic medical records. All laboratory results were produced from a centralized laboratory of Tongji Hospital using standard methods periodically recalibrated against the reference material. Mean arterial pressure was calculated by adding 1/3 of systolic blood pressure to 2/3 times diastolic blood pressure.

### 2.4. Definition of Exposures

The CAPA-LM equation pair was the default method for assessing SPS unless stated otherwise, by using the definition of eGFRcys < 70% of eGFRcr at baseline as previously reported [16, 21]. Corresponding equations were given below:

- The Caucasian Asian Pediatric Adult (CAPA) equation:

(1) $$\begin{array}{c} \text{eGFR}=130\times {\text{cysC}}^{-1.069}\times {\text{age}}^{-0.117}-7. \end{array}$$

(ii) The revised Lund-Malmö (LMrev) equation:

(2) $$\begin{array}{c} \text{eGFR}=e^{X-0.0158\times \text{age}+0.438\times \ln\left(\text{age}\right)}, \end{array}$$

where for females with creatinine < 150 *μ*mol/L, *X* is calculated as

(3) $$\begin{array}{c} X=2.50+0.0121\times \left(150-\text{creatinine}\right), \end{array}$$

for females with creatinine ≥ 150 *μ*mol/L, *X* is calculated as

(4) $$\begin{array}{c} X=2.50-0.926\times \ln\left(\text{creatinine}/150\right), \end{array}$$

for males with creatinine < 180 *μ*mol/L, *X* is calculated as

(5) $$\begin{array}{c} X=2.56+0.00968\times \left(180-\text{creatinine}\right), \end{array}$$

for males with creatinine ≥ 180 *μ*mol/L, X is calculated as

(6) $$\begin{array}{c} X=2.56-0.926\times \ln\left(\text{creatinine}/180\right). \end{array}$$

However, in sensitivity analyses, positive results were confirmed by examining the more relaxed CKD-EPI definition for diagnosis of SPS. Detailed equations are listed as follows:

- The cystatin C-based CKD-EPI (CKD-EPIcys) equation:

1. For females with cystatin C ≤ 0.8 mg/L,

(7) $$\begin{array}{c} \text{eGFR}=133\times {\left(\text{cysC}/0.8\right)}^{-0.499}\times 0.996^{\text{age}}\times 0.932 \end{array}$$

(2) For females with cystatin C > 0.8 mg/L,

(8) $$\begin{array}{c} \text{eGFR}=133\times {\left(\text{cysC}/0.8\right)}^{-1.328}\times 0.996^{\text{age}}\times 0.932 \end{array}$$

(3) For males with cystatin C ≤ 0.8 mg/L,

(9) $$\begin{array}{c} \text{eGFR}=133\times {\left(\text{cysC}/0.8\right)}^{-0.499}\times 0.996^{\text{age}} \end{array}$$

(4) For males with cystatin C > 0.8 mg/L,

(10) $$\begin{array}{c} \text{eGFR}=133\times {\left(\text{cysC}/0.8\right)}^{-1.328}\times 0.996^{\text{age}} \end{array}$$

(ii) The creatinine-based CKD-EPI (CKD-EPIcr) equation:

1. For females with creatinine ≤ 0.7 mg/dL,

(11) $$\begin{array}{c} \text{eGFR}=144\times {\left(\text{creatinine}/0.7\right)}^{-0.329}\times 0.993^{\text{age}} \end{array}$$

(2) For females with creatinine > 0.7 mg/dL,

(12) $$\begin{array}{c} \text{eGFR}=144\times {\left(\text{creatinine}/0.7\right)}^{-1.209}\times 0.993^{\text{age}} \end{array}$$

(3) For males with creatinine ≤ 0.9 mg/dL,

(13) $$\begin{array}{c} \text{eGFR}=141\times {\left(\text{creatinine}/0.9\right)}^{-0.411}\times 0.993^{\text{age}} \end{array}$$

(4) For males with creatinine > 0.9 mg/dL,

(14) $$\begin{array}{c} \text{eGFR}=141\times {\left(\text{creatinine}/0.9\right)}^{-1.209}\times 0.993^{\text{age}} \end{array}$$

### 2.5. Assessment of Outcomes

Medical records were screened, and all the outpatient and in-hospital creatinine results were exported from the clinical examination database till February 18th, 2022. ESRD referred to eGFR ≤ 15 mL/min/1.73 m^2^ or the initiation of renal replacement therapy. Severe eGFR decline was defined as stable serum creatinine doubling or ≥50% eGFRcr decline compared with baseline [22, 23]. For consolidation of our outcomes as well as ensuring the identification to be less biased by human selection or possible omission, a semiautomatic procedure was employed by first screening the creatinine lists using EXCEL algorithm for matching of outcome definition, and selected patients were further inspected manually by checking the creatinine lists and medical records to avoid transient creatinine bump and ensure a permanent functional loss. For all analyses, the follow-up period referred to the interval between the baseline visit and the last visit when creatinine was determined or the occurrence of the outcome of interest, whichever came first. Only eGFRcr estimated by the CKD-EPIcr equation were used to set baseline reference values and in later follow-up assessments.

### 2.6. Statistical Analyses

Categorical variables were represented as number (percentage). Continuous variables were either represented as the mean ± standard deviation when normally distributed or as median (25th~75th interquartile value) otherwise. An independent *t*-test or Mann–Whitney test was used according to data distribution to compare continuous variables. A chi-square test was conducted to compare nominal variables. Ordinal variables were compared using the Mann–Whitney test.

Kidney survival was analyzed using Kaplan-Meier plots followed by a log-rank test. Hazard ratios (HRs) and 95% confidence interval (95% CI) were calculated using Cox regression. Variables significantly associated with outcomes were adjusted in a stepwise manner: Model 1 was adjusted for basic demographics and anthropometrics—age, sex, and MAP (mean arterial blood pressure); Model 2 was further adjusted for follow-up treatments—ACEi/ARB, glucocorticoids, and immunosuppressants; Model 3 was further adjusted for kidney pathology—presence of glomerulosclerosis, crescents, and pathology diagnosis; Model 4 was further adjusted for laboratory results—baseline eGFR, bicarbonate, blood urea nitrogen, uric acid, total cholesterol, serum potassium, natrium, chloride, calcium, phosphate, hemoglobin, albumin, fibrinogen, and lgUALB (log value of urine albumin concentration). To minimize the possibility of overfitting, SPS was fitted using Enter method in block 1 followed by covariables fitted in block 2 using Forward LR (likelihood ratio) method. Urine albumin concentration was log transformed in Cox regression to approximate normal distribution.

Missing values were omitted in baseline description and group comparison where total number of patients with complete records is shown. However, in Cox regression, an imputed dataset where missing values were replaced by median values of the overall population was used [20]. If the main exposure reached statistical significance in the fully adjusted model, several sensitivity analyses would be performed by (1) using the SPS calculated by the CKD-EPI method (SPSCKD-EPI), (2) using continuous eGFRcys/eGFRcr ratio calculated by the CAPA-LM method as independent variable, and (3) using continuous eGFRcys/eGFRcr ratio calculated by the CKD-EPI method as independent variable. Subgroup analyses were conducted with respect to biopsy diagnoses and sex.

Double-sided *P* values < 0.05 were considered statistically significant. Patients' preselection procedure for determining outcomes, as well as data sorting and preprocessing was performed using Microsoft EXCEL (Redmond, WA. United States). All statistical calculations were performed using SPSS 26.0.0.0 (Chicago, IL, USA, IBM SPSS Statistics). Plots were drawn using R version 4.1.1 (R Project for Statistical Computing) with R packages survival and survminer loaded.

## 3. Results

### 3.1. Baseline Characteristics

We performed the patient selection procedure as shown in Figure 1, and detailed baseline characteristics and follow-up treatments are listed in Table 1. The median age was 37 years, and 51% were female. The final sample was composed of the IgAN subpopulation (*n* = 414, 77%) and the MN subpopulation (*n* = 122, 23%). The IgAN subpopulation comprised more female patients, were younger, and had higher creatinine and blood pressure, more pronounced kidney pathology with respect to glomerulosclerosis and crescent formation, and severer hematuria, whereas the MN patients had more prevalent glucocorticoids and immunosuppressant usage in the follow-up period, thicker basement membrane, higher blood cholesterol and fibrinogen, lower blood albumin, and more abundant urine albumin secretion.

We observed 44 patients (8%) possessing SPS in our overall population. Although the prevalence did not differ significantly between the IgAN (7%) and MN (12%) patients, the eGFRcys/eGFRcr ratio was significantly higher among IgAN patients compared with the MN population. Also, prevalence of SPS was significantly higher in male patients than in female patients (12% in men vs. 5% in women). Moreover, it is worth noting that the CKD-EPIcr equation overestimated GFR by around 5~10 mL/min/1.73 m^2^ compared to the LMrev equation (median eGFR: 95 mL/min/1.73 m^2^ by CKD-EPIcr vs. 84 mL/min/1.73 m^2^ by LMrev), whereas the two cystatin C-based equations performed similarly (median eGFR: 76 mL/min/1.73 m^2^ by CKD-EPIcys; 73 mL/min/1.73 m^2^ by CAPA). These unparallel differences caused the assessment of prevalence to be much high once the CKD-EPI formulae were used to determine SPS (95 patients with SPS_CKD-EPI_, 18%).

When comparing patients with and without SPS, we found those with SPS had significantly higher serum fibrinogen and lower albumin in the overall population. In subgroup analyses, creatinine level was higher and glomerulosclerosis was more common in SPS patients than in non-SPS ones among the IgAN subgroup; in MN subpopulation, a tendency of more urine albumin concentration in SPS patients than non-SPS ones was noted with a marginal significance (*P* = 0.088). As expected, serum cystatin C level was higher and both eGFRcys and eGFRcys/eGFRcr ratio were lower among all groups.

### 3.2. Analysis of ESRD

During the follow-up period of 27.7 months on average, 24 patients progressed to ESRD, including 21 patients with IgAN and 3 with MN.

The overall incidence rate of ESRD was 19.4 per 1000 person years. The presence of SPS increased the incidence rate of ESRD by 4.7-fold, from 15.6 per 1000 person years in the non-SPS group to the 73.3 per 1000 person years in the SPS population. In subgroup analyses, we found the fold change of ESRD incidence by the presence of SPS was the profoundest in female patients (13.9-fold) and was the mildest in male patients (2.2-fold). This was paralleled with the survival analyses (shown in Figures 2(a)–2(c)) showing a significant risk of SPS for ESRD occurrence in female but not male patients. However, although the fold change of ESRD incidence was higher MN subpopulation (6.9-fold) than in IgAN cohort (4.4-fold), survival analyses showed significant effect only in the IgAN but not the MN group, possibly owning to insufficient sample size in the MN group.

Moreover, after adjusting a variety of possible confounding factors, including demographics and anthropometrics (age, sex, and MAP), follow-up treatments (ACEi/ARB, glucocorticoids, and immunosuppressants), kidney pathology (crescents, glomerulosclerosis), and laboratory results (eGFR, urine albumin, etc.) as listed in Table 2, the hazard ratio of SPS for ESRD only remained significant in the IgAN group (HR 8.35, 95% CI: 2.10~33.26).

### 3.3. Analysis of Severe eGFR Decline

Automatic algorithm selected a total of 44 patients fulfilling the requirements for doubling of serum creatinine or loss of more than 50% eGFR. After carefully screening each patients' creatinine lists and medical records, we excluded 8 patients with transient eGFR decline and postponed the occurrence of severe eGFR decline by 39.9 months for one patient (the former was transient but the latter was a permanent loss) and finally determined 36 patients who had experienced severe eGFR decline in our follow-up.

The pattern of influence of SPS on occurrence of severe eGFR decline was somewhat similar to that seen in ESRD, with the fold increasement which was much higher in women than in men (6.6-fold vs. 3-fold). Of note, the fold increasement was the highest in MN patients (7.6 folds), which corresponds to the highest hazard ratio in Cox regression before adjustment. In IgAN patients, the presence of SPS brought about a 3.5-fold increasement of incidence of severe eGFR decline. Survival plots (shown in Figures 2(d)–2(h)) revealed significant correlation with outcomes in all groups, which also persisted after full multivariable adjustments in Cox regression except in the IgAN group (Table 3).

### 3.4. Sensitivity Analyses

In sensitivity analysis 1, the CKD-EPI equations identified more people (95 patients with all the 44 patients in previous SPS definition) with possibly milder situation due to the looser standard. Consequently, hazard ratio decreased in all settings and significant result only maintained in female patients after full adjustment with respect to the relationship between SPS and severe eGFR decline. Furthermore, we also tested the correlation between the eGFRcys/eGFRcr ratio calculated by both the CKD-EPI and the CAPA-LM methods and relevant outcomes. Still, only in female patients a higher eGFRcys/eGFRcr ratio was protective for eGFR decline after adjustments (Table 4).

## 4. Discussion

In this study, we investigated the prevalence of SPS in biopsy-proven IgAN and MN patients and assessed its association with kidney outcomes. SPS greatly increased the incidence rates of ESRD and severe eGFR decline. However, only in female patients the association between SPS and severe eGFR decline was statistically significant after multivariable adjustment and sensitivity analyses. Thus, our study suggests SPS as a potential risk factor for disease progression in female patients with kidney diseases.

The association of cystatin C with cardiovascular or renal outcomes have been discovered for a long time, and the predictive value of cystatin C for adverse clinical outcomes is not only superior to creatinine [24–27] but also exceeds that could be solely explained by mGFR [28, 29]. The proposal of SPS offers a reasonable explanation to this phenomenon. The adverse effects of SPS are based on two pathophysiological changes: (1) disrupted endothelial function and (2) the accumulation of low-molecular-weight proteins. Initially, the insight of SPS was gained from women in late-pregnancy, especially those with preeclampsia [9]. Steady or elevated cystatin C was observed in these patients accompanied by contrary changes of increased mGFR and reduced creatinine [30, 31]. Concurrent increase of molecules with similar size to cystatin C, i.e., beta-trace protein and beta2-microglobulin, was also noted [9]. Furthermore, markers related to NO metabolism such as Arg/ADMA ratio were found to diminish significantly [32]. All these facts point to dysregulated endothelial function, and it was hypothesized that swelling of glomerular endothelial cells causes shrinkage of glomerular filtration pores, which pose greater problem to filtration of relatively larger molecules [12]. Besides, thickening of glomerular filtration barrier leading to increased filtration length might also result in SPS as shown in diabetic nephropathy [10]. However, most theories mentioned above are still in the hypothetical stage, since few evidences directly observed the proposed morphological changes in basement membrane. Our study was the first one to carefully examining this syndrome in a group of patients with full kidney biopsy. Nonetheless, we only gained our information on kidney pathology from past biopsy records. We did not observe a significant difference in the prevalence of basement membrane thickening between SPS and non-SPS patients. Since only results from optical microscopy were available, we cannot assess the ultrastructure of kidney such as the basement barrier pores. Despite the above limitedness, some clues between SPS and kidney pathology was gained: first, in IgAN patients, the presence of SPS was associated with the occurrence of glomerulosclerosis; secondly, as a disease where basement membrane was deeply involved, although the prevalence of SPS in MN patients was not statistically higher than IgAN patients, the significantly lower eGFRcys/eGFRcr ratio in MN patients compared to those with IgAN might hint possible correlation with basement membrane abnormalities. More direct evidences are needed to clarify the underlying pathophysiology of SPS.

Previous researches unveiled the existence of SPS in diverse populations with varying prevalence rate from 0.2% to 36%, and the occurrence of SPS is irrelevant to conventional GFR measured by small molecules, reflecting the role of SPS as a formerly unrecognized type of renal dysfunction [11]. The selectively accumulated proteins consist of cytokines, hormones, growth factors, and signaling peptides, many of which have proatherosclerotic effects as corroborated by proteomic studies [33, 34]. Accordingly, most studies concerning SPS demonstrated adverse cardiovascular endpoints [19, 20, 35]. However, few studies conducted so far related SPS to renal outcomes, and our study was the first one to our knowledge that assess the relationship between SPS and ESRD or eGFR decline in patients suffering kidney diseases of known pathological diagnoses.

There is no consensus regarding the cut-off value for defining SPS. Both 60% and 70% eGFRcys/eGFRcr ratio have been used in previous studies [14, 15, 17]. Continuous ratio has also been explored in some researches where the above cut-off values identified few patients [19, 20, 36]. We chose the cut-off value of 70% as previous studies have shown that adverse effects already come into play in early stage when eGFRcys/eGFRcr ratio falls to 85% or 90% [16, 18].

The major difference between the CKD-EPI and CAPA-LM standards lay in the higher eGFRcr computed by the CKD-EPIcr than the LMrev equation. This resulted in lower eGFRcys/eGFRcr ratio by the CKD-EPI equations compared to the CAPA-LM equations, which led to greater proportion of patients classified as SPS. In other words, the CAPA-LM definition represents a stricter criterion for SPS classification that identifies patients with more advanced pathophysiological changes. This judgment could be verified by the fact that all the 44 afflicted patients by SPSCAPA-LM were also included in the 95 patients with SPSCKD-EPI. The hazard ratios were generally greater, and statistical significances were more pronounced by SPSCAPA-LM compared to that of SPSCKD-EPI, which were also present in other studies involving both definitions [15, 17, 18]. This indicates the pathophysiology of SPS as a continuous spectrum, with more harmful effects caused by more severe pathophysiological changes.

Although incidence rates of both ESRD and severe eGFR decline were dramatically elevated under SPS, we could only demonstrate significant effect concerning eGFR decline after multivariable adjustment in female patients. Due to limited follow-up duration of around one and a half year by median, ESRD happened in only 24 patients of our sample. Thus, insufficient sample size might account for our inability to get a significant result. However, since doubling of creatinine or more than 50% eGFR decline have been established as reliable surrogate markers for final ESRD [22, 23], we are convinced that significant hazard of SPS on eGFR decline would transfer into the future development for ESRD, which can be proved with larger datasets or longer follow-up.

Sex difference was observed in our study, as the prevalence of SPS was lower but the HR was significant in women compared to men. Sex-related difference has been reported in some researches: a lower eGFRcys/eGFRcr ratio was shown to be hazardous in the development of first-ever myocardial infarction [19] and aortic stenosis requiring surgery [20] only in women but not in men. However, the present study was the first one to our knowledge reporting sex differences of SPS regarding renal outcomes. Part of the causes might lie in sex-related differences in blood biomarkers, as both muscle mass and blood creatinine are higher in men compared to women [6], which possibly result in differential effects when the same cut-off value is used to diagnose SPS. This difference was partially adjusted when sex factor was incorporated into the estimation equations of eGFR. Furthermore, in sensitivity analyses, we investigated the effects of the continuous factor eGFRcys/eGFRcr on renal prognosis in different sexes separately, and only in women the ratio had a meaningful prognostic value. As sex differences existed in many situations such as cancer risk [37] and cardiovascular complications [38] and molecular pathways mediating sex difference in response to kidney injury has been reported [39], it was reasonable that sex difference was not only due to inappropriate selection of cut-off value, but more likely resulted from greater vulnerability to various accumulated substances of SPS in women than in men.

Even if cystatin C has many advantages in clinics, special caution must be paid to non-renal influences of cystatin C, which might deviate the true level of eGFRcys/eGFRcr ratio and cause false classification of SPS. One of the most prevalent nonrenal influences in patients with kidney diseases is the use of glucocorticoids, which is frequently prescribed in immunologic kidney diseases and causes abnormal elevation of cystatin C [40–42]. Another important factor is thyroid disorders [43]. Practical solutions to identify SPS in these patients might be achieved by replacing or supplementing cystatin C with other low-molecular-weight proteins sharing similar characteristics but different response to glucocorticoids, e.g., beta-trace protein [9]. However, reliable methods need further validation to confirm their effectiveness.

Our study has both limitations and strengths. The major limitation is the retrospective observational design, which prohibited us to test causal relationships. Second, limited sample size not only restricted the statistical power to gain significant results but also diminished the reliability of our conclusion. However, as we employed a group of sensitivity analyses, we are convinced to the validity of our results. Further, mGFR is not measured in our study. Using eGFRcr to approximate mGFR suffered from the risk of non-renal influences of creatinine, for example, sarcopenia. Though lack of parameters such as body mass index prevented us to rule out the risk, we believe it is not very likely due to our SPS group had higher creatinine value at baseline compared to the non-SPS patients. The primary strength of our study relates to the clearly defined pathologic changes diagnosed by biopsy, which have not been studied before and the homogenous pathologic background reduces possible confounding factors. Second, we adjusted various potential factors in multivariable models encompassing basic demographics, anthropometric measurements, important medication, and laboratory parameters. Third, sensitivity analyses listed above made our results more convincing.

## 5. Conclusions

In conclusion, we investigated the incidence rates and clinical consequences of SPS in patients with IgAN or MN and found significant association between SPS and eGFR decline in female patients. Further studies are needed to verify the link between SPS and renal outcomes in larger prospective cohorts concerning diverse populations.

## Figures and Tables

**Figure 1:** Flow chart of the patient selection procedure.

**Figure 2:** Kaplan-Meier plots of ESRD and severe eGFR decline among patients with and without SPS depicting the relationship between (a) ESRD and SPS in overall population; (b) ESRD and SPS in IgAN subgroup; (c) ESRD and SPS in female patients; (d) severe eGFR decline and SPS in overall population; (e) severe eGFR decline and SPS in IgAN subgroup; (f) severe eGFR decline and SPS in MN subgroup; (g) severe eGFR decline and SPS in female patients; and (h) severe eGFR decline and SPS in male patients. ESRD: end-stage renal disease; SPS: shrunken pore syndrome; IgAN: IgA nephropathy; MN: membranous nephropathy.

**Table 1:** Baseline characteristics of the study population.

Population	Overall	IgAN (*n* = 414)		MN (*n* = 122)	
	Total (*n* = 536)	Non-SPS (*n* = 384, 93%)	SPS (*n* = 30, 7%)	Non-SPS (*n* = 108, 88%)	SPS (*n* = 14, 12%)
Characteristics					
Age, years^d^	37 (27~48)	33 (26~44)	34 (27~43)	50 (41~59)	48 (44~55)
Women, no. (%)^c,d^	274 (51%)	220 (57%)	12 (40%)	40 (37%)	2 (14%)
Mean arterial BP (mmHg), *n* = 523^d^	97 ± 13	96 ± 13	100 ± 13	99 ± 13	100 ± 11
Medication∗					
ACEi or ARB, no. (%)	214 (40%)	159 (41%)	14 (47%)	37 (34%)	4 (29%)
Glucocorticoids, no. (%)^d^	316 (59%)	215 (56%)	19 (63%)	72 (67%)	10 (71%)
Immunosuppressants, no. (%)^d^	129 (24%)	72 (19%)	4 (13%)	45 (42%)	8 (57%)
Renal pathology					
Glomerulosclerosis, no. (%)^a,d^	393 (73%)	299 (78%)	28 (93%)	59 (55%)	7 (50%)
Percent of crescents^d^					
C0 (0%)	288 (54%)	163 (42%)	14 (47%)	99 (92%)	12 (86%)
C1 (<25%)	197 (37%)	174 (45%)	12 (40%)	9 (8%)	2 (14%)
C2 (≥25%)	51 (10%)	47 (12%)	4 (13%)	0 (0%)	0 (0%)
Basement membrane thickening^d^					
Without thickening, no. (%)	354 (66%)	323 (84%)	28 (93%)	3 (3%)	0 (0%)
Segmental thickening, no. (%)	86 (16%)	55 (14%)	2 (7%)	26 (24%)	3 (21%)
Diffuse thickening, no. (%)	96 (18%)	6 (2%)	0 (0%)	79 (73%)	11 (79%)
Laboratory					
Creatinine (*μ*mol/L)^a,d^	80 (64~104)	80 (63~109)	94 (79~123)	75 (63~89)	72 (62~94)
eGFR (CKD-EPIcr) (mL/min/1.73 m^2^)	95 (69~112)	93 (64~116)	82 (53~100)	98 (79~108)	102 (85~110)
eGFR (LMrev) (mL/min/1.73 m^2^)^d^	84 (64~98)	82 (61~98)	75 (51~87)	86 (72~95)	90 (78~101)
Cystatin C (mg/L)^a,b,c^	1.1 (0.9~1.3)	1.0 (0.8~1.3)	1.5 (1.3~2.2)	1.0 (0.8~1.2)	1.3 (1.2~1.6)
eGFR (CKD-EPIcys) (mL/min/1.73 m^2^)^a,b,c^	76 (58~100)	78 (58~102)	47 (28~61)	80 (65~100)	58 (46~65)
eGFR (CAPA) (mL/min/1.73 m^2^)^a,b,c^	73 (56~94)	76 (58~96)	48 (30~59)	76 (63~93)	57 (45~62)
eGFRcys/eGFRcr (CKD-EPI)^a,b,c,d^	0.85 (0.74~0.96)	0.87 (0.78~0.98)	0.59 (0.52~0.62)	0.83 (0.76~0.97)	0.59 (0.53~0.64)
eGFRcys/eGFRcr (CAPA-LM)^a,b,c,d^	0.92 (0.81~1.05)	0.96 (0.86~1.08)	0.66 (0.59~0.68)	0.89 (0.82~1.03)	0.63 (0.57~0.66)
Total cholesterol (mmol/L), *n* = 523^d^	4.47 (3.83~5.43)	4.26 (3.72~4.84)	4.31 (3.71~5.18)	6.07 (5.14~7.80)	6.92 (5.34~8.85)
Albumin (g/L), *n* = 513^c,d^	39.8 (34.2 ~43.3)	40.8 (38.7 ~44.1)	41.1 (36.4~42.7)	29.6 (24.3~35.6)	27.2 (21.4~31.5)
Hemoglobin (g/dL), *n* = 518	13.2 ± 1.8	13.1 ± 1.8	12.9 ± 2.1	13.6 ± 2.0	14.2 ± 9.3
Fibrinogen (g/L), *n* = 485^c,d^	3.5 (2.9~4.4)	3.3 (2.8~3.9)	3.5 (3.0~4.4)	4.7 (4.0~5.8)	4.5 (4.0~6.2)
Urine albumin (g/L), *n* = 483^d^	0.6 (0.2~1.7)	0.5 (0.2~1.0)	0.5 (0.1~1.0)	2.7 (0.8~5.2)	4.4 (2.2~6.5)
Hematuria^d^					
Negative (-), no. (%)	35 (6%)	24 (6%)	3 (10%)	7 (6%)	1 (7%)
Semi-positive (±), no. (%)	36 (7%)	23 (6%)	3 (10%)	8 (7%)	2 (14%)
1+, no. (%)	59 (11%)	28 (7%)	2 (7%)	27 (25%)	2 (14%)
2+, no. (%)	144 (27%)	95 (25%)	4 (13%)	39 (36%)	6 (43%)
3+, no. (%)	251 (47%)	208 (54%)	16 (53%)	24 (22%)	3 (21%)

SPS: shrunken pore syndrome; CKD-EPI: Chronic Kidney Disease Epidemiology Collaboration equations for creatinine-based (CKD-EPIcr) or cystatin C-based (CKD-EPIcys) eGFR estimation; CAPA: Caucasian Asian Pediatric Adult equation; LM or LMrev: revised Lund-Malmö equation; IgAN: IgA nephropathy; MN: membranous nephropathy; BP: blood pressure; ACEi: angiotensin converting enzyme inhibitors; ARB: angiotensin receptor blockers; BUN: blood urea nitrogen. ^∗^Medication represents the usage of corresponding drugs (RAASi, glucocorticoids, or immunosuppressants) in follow-up since baseline. a, b, and c represent statistically significant differences between non-SPS and SPS patients among the IgAN, MN, and the overall population, respectively, while d denotes significant difference between the IgAN and MN patients.

**Table 2:** Cox regression analysis for ESRD according to the presence or absence of SPS. The number of event/sample population and percentage are displayed in each group analyzed.

Groups (events/no.)	Overall (24/536)		Male (15/262)		Female (9/274)		IgAN (21/414)		MN (3/122)	
Models	HR (95% CI)	*P*	HR (95% CI)	*P*	HR (95% CI)	*P*	HR (95% CI)	*P*	HR (95% CI)	*P*
Unadjusted	3.91 (1.45, 10.55)	0.01	2.39 (0.67~8.59)	0.18	8.59 (1.67~44.27)	0.01	3.50 (1.17~10.51)	0.02	6.61 (0.60~73.07)	0.12
Model 1	3.85 (1.42, 10.41)	0.01	2.69 (0.74~9.75)	0.13	8.59 (1.67~44.27)	0.01	3.60 (1.19~10.85)	0.02	6.61 (0.60~73.07)	0.12
Model 2	3.14 (1.11, 8.88)	0.03	2.40 (0.66~8.70)	0.18	8.59 (1.67~44.27)	0.01	2.54 (0.75~8.60)	0.13	6.61 (0.60~73.07)	0.12
Model 3	3.66 (1.24, 10.84)	0.02	2.74 (0.75~10.02)	0.13	8.59 (1.67~44.27)	0.01	3.30 (0.89~12.17)	0.07	6.61 (0.60~73.07)	0.12
Model 4	1.70 (0.47, 6.13)	0.42	6.39 (0.92~44.10)	0.06	0.21 (0.02~2.50)	0.22	8.35 (2.10~33.26)	0.003	Not convergent	/

Model 1 was adjusted for basic demographics—age, sex, and MAP (mean arterial blood pressure); Model 2 was further adjusted for follow-up treatments—ACEi/ARB, glucocorticoids, and immunosuppressants; Model 3 was further adjusted for kidney pathology—presence of glomerulosclerosis, crescents, and pathology diagnosis; Model 4 was further adjusted for laboratory results—baseline eGFR, bicarbonate, blood urea nitrogen, uric acid, total cholesterol, serum potassium, natrium, chloride, calcium, phosphate, hemoglobin, albumin, fibrinogen, and lgUALB (log value of urine albumin concentration). ESRD: end-stage renal disease; SPS, shrunken pore syndrome; HR: hazard ratio; 95% CI: 95% confidence interval; IgAN: IgA nephropathy; MN: membranous nephropathy.

**Table 3:** Cox regression analysis for severe eGFR decline according to the presence or absence of SPS. The number of event/sample population and percentage are displayed in each group analyzed.

Groups (events/no.)	Overall (36/536)		Male (20/262)		Female (16/274)		IgAN (30/414)		MN (6/122)	
Models	HR (95% CI)	*P*	HR (95% CI)	*P*	HR (95% CI)	*P*	HR (95% CI)	*P*	HR (95% CI)	*P*
Unadjusted	3.45 (1.49~7.96)	0.004	3.01 (1.08~8.39)	0.04	5.12 (1.12~23.44)	0.04	2.70 (1.02~7.17)	0.05	6.62 (1.20~36.45)	0.03
Model 1	3.48 (1.51~8.02)	0.003	3.26 (1.17~9.08)	0.02	5.12 (1.12~23.44)	0.04	2.93 (1.10~7.79)	0.03	6.62 (1.20~36.45)	0.03
Model 2	3.50 (1.50~8.15)	0.004	3.03 (1.09~8.44)	0.03	10.30 (1.93~54.92)	0.01	2.87 (1.07~7.73)	0.04	5.25 (0.92~30.13)	0.06
Model 3	3.73 (1.56~8.91)	0.003	2.45 (0.83~7.23)	0.10	12.88 (2.33~71.23)	0.003	3.97 (1.42~11.10)	0.01	5.25 (0.92~30.13)	0.06
Model 4	2.76 (1.03~7.37)	0.043	10.29 (2.52~41.93)	0.001	7.54 (1.28~44.32)	0.02	2.42 (0.65~9.00)	0.19	84.98 (1.39~5181.14)	0.03

Model 1 was adjusted for basic demographics—age, sex, and MAP (mean arterial blood pressure); Model 2 was further adjusted for follow-up treatments—ACEi/ARB, glucocorticoids, and immunosuppressants; Model 3 was further adjusted for kidney pathology—presence of glomerulosclerosis, crescents, and pathology diagnosis; Model 4 was further adjusted for laboratory results—baseline eGFR, bicarbonate, blood urea nitrogen, uric acid, total cholesterol, serum potassium, natrium, chloride, calcium, phosphate, hemoglobin, albumin, fibrinogen, and lgUALB (log value of urine albumin concentration). SPS: shrunken pore syndrome; HR: hazard ratio; 95% CI: 95% confidence interval; IgAN: IgA nephropathy; MN: membranous nephropathy.

**Table 4:** Sensitivity analyses for association between ESRD or severe eGFR decline and SPS by multivariable Cox regression analysis. All the analyses were adjusted for confounders as model 4 in previous tables.

Setting	eGFR decline-all		eGFR decline-male		eGFR decline-female		eGFR decline-MN		ESRD-IgAN	
Analyses	HR (95% CI)	*P*	HR (95% CI)	*P*	HR (95% CI)	*P*	HR (95% CI)	*P*	HR (95% CI)	*P*
Analysis 1	1.87 (0.86~4.06)	0.12	2.21 (0.73~6.72)	0.16	3.71 (1.10~12.50)	0.04	Not convergent	/	0.79 (0.20~3.14)	0.74
Analysis 2	0.19 (0.03~1.07)	0.06	3.93 (0.36~42.95)	0.26	0.02 (0.001~0.52)	0.002	0.21 (0.01~6.23)	0.37	0.88 (0.08~9.94)	0.92
Analysis 3	0.42 (0.06~2.96)	0.38	4.26 (0.37~48.90)	0.24	0.01 (0.000~0.44)	0.02	0.24 (0.01~8.13)	0.43	1.22 (0.10~14.11)	0.88

Analysis 1 used the SPS classification calculated by CKD-EPI equations (SPSEPI); Analysis 2 used continuous eGFRcys/eGFRcr ratio by CAPA-LM equations; Analysis 3 used continuous eGFRcys/eGFRcr ratio by CKD-EPI equations. ESRD: end-stage renal disease; SPS: shrunken pore syndrome; HR: hazard ratio; 95% CI: 95% confidence interval; CKD-EPI: Chronic Kidney Disease Epidemiology Collaboration equations; CAPA: Caucasian Asian Pediatric Adult equation; LM: revised Lund-Malmö equation; IgAN: IgA nephropathy; MN: membranous nephropathy.

## Data Availability

The raw data used to support the findings of this study are available from the corresponding authors upon request.
